The article "18F-labeled Dimer-Sansalvamide A Cyclodecapeptide: A Novel Diagnostic Probe to Discriminate Pancreatic Cancer from Inflammation in a Nude Mice Model" was published in 2022. Journal: J Cancer.

# ^18^F-labeled Dimer-Sansalvamide A Cyclodecapeptide: A Novel Diagnostic Probe to Discriminate Pancreatic Cancer from Inflammation in a Nude Mice Model

**DOI:** 10.7150/jca.69710

**Published:** 2022-03-21

**Authors:** Xiaohui Wang, Jun Zhang, Zhijian Han, Liheng Ma, Yumin Li

**Affiliations:** 1 Medical Imaging Department, First Affiliated Hospital of Guangdong Pharmaceutical University, Guangzhou, 510080, China.; 2 Department of Nuclear Medicine, Taizhou People's Hospital, Taizhou, 225300, China.; 3 Molecular Imaging Center, Department of Radiology, Keck School of Medicine, University of Southern California, Los Angeles, 90033, USA.; 4 Key Laboratory of Digestive System Tumors of Gansu Province, Lanzhou University Second Hospital, Lanzhou, 730000, China.

**Keywords:** Positron emission tomography (PET), heat shock protein 90 (Hsp90), pancreatic cancer, Dimer-Sansalvamide A cyclodecapeptide, ^18^F labeling

## Abstract

Early detection of pancreatic cancer has been a long-standing challenge. Inflammatory mass is the main source of false-positive findings in ^18^F-labeled fluorodeoxyglucose (^18^F-FDG) positron emission tomography / computed tomography (PET/CT). Heat shock protein 90 (Hsp90) is an established biomarker overexpressed in pancreatic cancer. We modified a Dimer-Sansalvamide A cyclodecapeptide by conjugating it with the bifunctional chelator NOTA (1,4,7-triazacyclononane-1,4,7-trisacetic acid), yielding ^18^F-NOTA-Dimer-Sansalvamide A cyclodecapeptide (^18^F-NOTA-Dimer-San A). The binding specificity of the probe was confirmed by *in vitro* cell uptake assays in Hsp90-positive PL45 pancreatic cancer cells. Hsp90 expression was imaged via MicroPET in pancreatic cancer xenografts and inflammation in mice. All of the mice received an intravenous injection of ^18^F-NOTA-Dimer-San A, and images were acquired at 1 and 2 hour time points. The novel probe demonstrated prominent tumor uptake in the pancreatic cancer xenografts (4.00 ± 0.88 %ID/g, 5.80 ± 0.94 %ID/g), and the inflammatory thigh showed minimal uptake (0.85 ± 0.01 %ID/g, 1.50 ± 0.20 %ID/g) at 1 and 2 hours after injection, respectively. The activity accumulation between the two groups was significantly different (*P* < 0.05), and the biodistribution data was consistent with the images. Moreover, immunohistochemistry (IHC) confirmed that the expression of Hsp90 was positive in PL45 pancreatic cancer but negative in the muscles next to the tumor and inflammatory muscles. We concluded that ^18^F-NOTA-Dimer-San A PET might allow non-invasive imaging for Hsp90 expression in tumors and has the potential to discriminate pancreatic cancer from inflammatory mass.

## Introduction

Pancreatic cancer is an intractable malignancy and is the seventh leading cause of global cancer deaths worldwide. However, its toll is higher in more developed countries 1. Despite advancements in the detection and management of pancreatic cancer, the 5-year survival rate still stands at 9% only. Overall survival has not improved over the past two decades. Surgery is only possible in around 20% of new cases, and 80% of patients have local progression or metastasis at the time of diagnosis 2-4.

Early detection of pancreatic cancer is difficult, and discriminating inflammatory changes of the pancreas from neoplastic change has been a long-standing challenge 5. The imaging techniques currently used, including ultrasound, magnetic resonance imaging (MRI), and computed tomography (CT), have various limitations, including the difficulty in discriminating between benign and malignant tumors. Positron emission tomography (PET) is a newly emerged modality, which can offer functional information of the disease and non-invasively detect the expression of indicative molecular targets in living subjects. ^18^F-fluorodeoxyglucose (^18^F-FDG), the analog of glucose, is currently the most widely used radiopharmaceutical in clinical oncology. Although the application of ^18^F-FDG PET in tumor detection, staging, and therapy evaluation is rapidly expanding, ^18^F-FDG is a non-specific tracer. The limitations of ^18^F-FDG PET in the diagnosis of pancreatic cancer mainly include possible false-negative results in hyperglycemia and possible false-positive results in inflammatory masses 5-9.

In the laboratory, great efforts have been made to detect pancreatic cancer accurately by molecular discrimination using specific highly expressed biomarkers 5. Due to the radiolabeling techniques, numerous radiopharmaceuticals, including peptide-based agents, have been developed, and early diagnosis of pancreatic cancer has been evaluated 7, 10-14.

Heat shock protein 90 (Hsp90) is a well-established oncogenic target. It is elevated in the majority of cancers, but is 6- to 7-fold higher in human pancreatic cancer than normal tissues 15. Hsp90 inhibitors selectively bind to Hsp90 and provoke apoptosis of cancer cells. It was confirmed that Hsp90 derived from cancer cells has a 100-fold higher binding affinity for 17-allylaminogeldanamycin (17-AAG), a Hsp90 inhibitor, than does Hsp90 from normal cells 16. Therefore, Hsp90 has become an attractive target in the field of cancer therapeutics and diagnostics 17, 18.

Sansalvamide A (San A), a natural product isolated from a marine fungus (*Fusarium ssp.*), exhibits significant antitumor ability at micromolar potency 19-22. Syntheses and evaluation of San A and its peptide analog have revealed that the analog has greater potency against human carcinoma than the natural depsipeptide 21, 23. It has been confirmed that San A and its derivatives are Hsp90 inhibitors that directly bind to Hsp90 and modulate the binding of Hsp90 with its client proteins, inducing cell apoptosis 23-25. At present, there are hundreds of San A derivatives, which have significant differences in the growth inhibition of cancer cells 21, 26, 27. By comparing the cytotoxicity of each compound, Dimer-Sansalvamide A cyclodecapeptide (Dimer-San A) exhibited excellent potency (IC_50_, 1-20 nM) in the inhibition of pancreatic cancer PL45 cells. For the first time ever, we selected a metallic PET isotope copper-64 (^64^Cu) to construct a PET probe ^64^Cu-Di-San A1 based on the potency of the peptide. ^64^Cu-labeled dimeric Sansalvamide A decapeptide has been successfully prepared for PET imaging of Hsp90 expression in PL45 pancreatic cancer mouse xenografts 28. However, in MicroPET imaging and biodistribution studies, we observed a relatively high accumulation and retention in mouse liver, which may be due to partial demetallation of ^64^Cu-1, 4, 7-triazacyclononane-N, N', N”-triacetic acid (NOTA) complexes in the mouse liver. Additionally, radiopharmaceutical ^64^Cu is expensive and not easily available. Fluorine-18 (^18^F) (β^+^, 511 KeV, 97%; t_1/2_ =110 min) offers ideal benefits over ^64^Cu. Based on the above factors, in this study, we labeled the Dimer-San A cyclodecapeptide with ^18^F, the most widely used radionuclide, and explored its value in the differential diagnosis of pancreatic cancer.

## Materials and methods

### General

All chemicals (reagent grade) were obtained from commercial suppliers and used without further purifcation. Dimer-San A was modified by conjugating with the bifunctional chelator, NOTA, which was purchased from Chinese Peptide Company (Hangzhou, China) with a purity of > 95%. Biotine-Dimer-San A peptide was also obtained from Chinese Peptide Company. Anti-hsp90α antibody was purchased from Abcam (Cambridge, UK), and 17-AAG was purchased from Thermo Fisher Scientifc, USA.

### Cell culture

PL45 pancreatic ductal adenocarcinoma cell line was obtained from the American Type Culture Collection (ATCC, Manassas, VA, USA) and maintained in Dulbecco's Modified Eagle's Medium (DMEM) supplemented with 10% fetal bovine serum (Thermo Fisher Scientifc, NY, USA). The cells were grown in 95% relative humidified atmosphere containing 5% CO_2_ at 37 °C.

### Cell immunofluorescence

PL45 cells (3-5 × 10^5^) were seeded in a confocal plate with 500 µL of culture medium and incubated for 24 hours at 37°C with 5% CO_2_. The cell culture medium was then removed, and the cells were rinsed 3 times using phosphate buffered saline (PBS). The cells were fixed using 400 µL of 4% paraformaldehyde (pH 7.4) for 20 minutes at room temperature (RT, ~20°C). Then 500 µL of 3% Bovine Serum Albumin (BSA) (Sigma-Aldrich Corp., St. Louis, MO, USA) was added and incubated for 30 minutes at RT for blocking. The cells were washed and then 250 µL of diluted anti-hsp90α antibody (1:250) or biotine-Dimer-San A peptide was added and incubated for 24 hours at 4°C. The cells were washed, and the desired concentration of the fluorescent-dye-labeled secondary antibody (Abcam, Cambridge, UK) or Cy5 labeled avidin (Vector Laboratories, Burlingame, CA, USA) was added and protected from light at RT for 60 minutes. The supernatant was discarded, and the cells were washed, then a drop of antifade mounting medium with DAPI (Vector Laboratories, Burlingame, CA, USA) was added and incubated for 45 minutes. The target antigen was visualized by confocal fluorescence microscopy Zeiss LSM 880 Airyscan (Carl Zeiss AG, Oberkochen, Germany).

### Bioactivity assay of NOTA-Dimer-San A

A 3-(4,5-Dimethylthiazol-2-yl)-2,5-Diphenyltetrazolium Bromide (MTT) (Thermo Fisher Scientifc, NY, USA) assay was used to test the bioactivity of NOTA-Dimer-San A cyclodecapeptide. PL45 cells (5000 cells) were seeded in a 96-well plate and incubated overnight. The culture medium was discarded, and 100 μL of different concentrations of NOTA-Dimer-San A (40000, 800, 160, 32, 6.4, 1.28 and 0.256 nM) or 17AAG (40000, 800, 160, 32, 6.4, 1.28 and 0.256 nM) were added to the wells. Each concentration was performed in triplicate, and the drug was incubated with the cells for 72 hours. Then 10 μL of MTT (5 mg/mL) was added into each well, incubated for 4 hours until a purple precipitate was visible, and then 100 μL of a detergent reagent was added and incubated until the crystal was dissolved. Finally, the optical density (proportional to the number of live cells) was assessed with a Synergy H1 Hybrid Reader (BioTek^®^ Instruments Inc., Winooski, Vermont, USA) at 570 nm. The cell viability (%) was calculated with GraphPad Prism 5.0 software (GraphPad Software Inc., San Diego, CA, USA).

### HPLC methods

The analytic and semi-preparative reversed phase high-performance liquid chromatography (HPLC) was performed on a Dionex Ultimate 3000 system (Thermo Fisher Scientifc, NY, USA). Semi-preparative reversed phase HPLC was performed using a Phenomenex Luna C18(2) reversed phase column (5 μm, 250×10 mm). The flow rate was 4 mL/min, with the mobile phase starting from 95% solvent A (0.1% trifluoroacetic acid (TFA) in water) and 5% solvent B (0.1% TFA in acetonitrile) to 100% solvent B at 20 min and remaining 100% solvent B for additional 4.5 min. The UV absorbance was monitored at 214 and 254 nm. The analytical HPLC was carried out using a Dionex Acclaim C18 reversed phase analytical column (5 μm, 250 × 4.6 mm). The flow rate was 1 mL/min with the mobile phase starting from 100% solvent A (0.1% TFA in water) to 100% solvent B (0.1% TFA in acetonitrile) at 15 min and remaining 100% solvent B for additional 5 min. The radioactivity was detected by a Ludlum 2200 single channel radiation detector (Ludlum Measurements Inc., Sweetwater, TX, USA).

### ^18^F-labeling of NOTA-Dimer-San A

The modified NOTA-Dimer-San A cyclodecapeptide was labeled with ^18^F in a two-step method, and the labeling reaction is summarized in Fig. 1. Firstly, 12-15 μL of 0.01 M AlCl_3_ and 5-10 μL of glacial acetic acid were added to a glass vial. Then 50-100 μL (555-740 MBq) Na^18^F was added and heated at 100°C for 10 minutes. Subsequently, 100-150 μg of NOTA-Dimer-San A peptide dissolved in 350-500 μL of acetonitrile and 40 μL of deionized water was added to the above vial. Finally, the reaction mixture was incubated at 100°C for 10 minutes and purifed by semi-preparative HPLC. The radioactive peak containing the ^18^F-NOTA-Dimer-San A peptide was collected and concentrated by rotary evaporation. The product was redissolved in 500 µL of PBS with 1% DMSO and passed through a 0.22-μm Millipore filter into a sterile vial for use in the following experiments.

### Octanol-water partition coefficient (log* P*_octanol/water_)

To determine the lipophilicity of the ^18^F-labeled NOTA-Dimer-San A, approximately 185 kBq ^18^F-NOTA-Di-San A was diluted in 500 μL of PBS, and an equal volume of octanol was added to obtain a binary phase system. After stirring in a vortex mixer for 1 minute, the two layers were separated by centrifugation (12500 rpm, 5 min). Three 100 μL samples were taken from each layer, and the radioactivity was measured by a γ-counter (PerkinElmer Wizard 2480 Automatic Gamma Counter) (PerkinElmer Singapore Pte Ltd, Singapore). The value was calculated as the mean ± standard deviation (SD).

### *In vitro* stability assay

The *in vitro* stability of ^18^F-NOTA-Dimer-San A was analyzed in PBS and mouse serum after purification by radio-HPLC at physiological temperature (37 °C) at 1 and 2 hour time points. Briefly, 3.7 MBq of ^18^F-NOTA-Dimer-San A was pipetted into 0.5 mL of PBS or mouse serum and incubated at 37 °C with gentle shaking. For the PBS study, an aliquot of the solution was directly taken at 1 and 2 hours after incubation, and the radiochemical purity was determined by reverse-phase analytical HPLC. For the mouse serum study, TFA was added to the mixture at 1 and 2 hours after incubation, and the soluble fraction was filtrated with a 0.22 μm filter. An aliquot of the solution was used to determine the radiochemical purity by reverse-phase analytical HPLC under an identical condition.

### *In vitro* cell uptake assay and blocking studies

PL45 cells were seeded into a 24-well plate at a density of 0.5 × 10^5^ cells per well and incubated overnight. Cells were rinsed twice with PBS, followed by the addition of 100 μL of ^18^F-NOTA-Dimer-San A (185 kBq) solution, and incubated for 15, 30, 60, 90, and 120 minutes at 37 °C. For the blocking study, PL45 cells were incubated as described above with 100 μL 17AAG (50 μM). After incubation, the supernatant was removed, and the cells were washed three times with PBS and lysed with 500 µL of 1 M NaOH. Finally, the cell lysate was collected in measurement tubes for counting with an automatic γ-counter. All experiments were performed twice with triple wells.

### Tumor xenografts and inflammation model establishment

All animal studies were performed according to the protocol approved by University of Southern California Institutional Animal Care and Use Committee (Los Angeles, CA, USA). Athymic nude mice (4-6 weeks, female) with a body weight of 22.6-32.9 g were ordered from Harlan (Livermore, CA, USA).

Tumor xenografts (n = 3) were generated by subcutaneous injection of 10 × 10^6^ PL45 cells resuspended in 50% PBS and 50% Matrigel Matrix (Corning, NY, USA) into the right shoulder of the mouse. The injected volume was 100-150 μL. The PL45 cells were allowed to grow until the tumor reached 100-300 mm^3^ in volume. Tumor growth was measured using caliper measurements in orthogonal dimensions.

The inflammation models were established as previously described by Van Waarde et al. 8. Briefly, 100 μL of turpentine was intramuscularly injected into the thigh of the left hind leg of another three mice, inducing the acute inflammatory reaction. After 24 hours, these inflammation models underwent MicroPET scans.

### Animal PET/CT image acquisition and analysis

All of the tumor- and inflammation-bearing mice were imaged in the prone position in the MicroPET scanner (Siemens, Munich, Germany). The mice were anesthetized with 2% isoflurane and injected with 5.55-7.4 MBq of the new radiotracer via the tail vein. Static scans were obtained for 5 minutes at 1 and 2 hours post-injection (pi). The images were reconstructed by a two-dimensional ordered-subsets expectation maximum (OSEM2D) algorithm. After each micro-PET scan, the regions of interest (ROIs) were drawn over the tumor, liver, kidneys, and inflamed muscle on decay-corrected whole-body coronal images using Inveon Research Workplace (IRW, Siemens, Munich, Germany) to obtain the imaging ROI-derived percentage injected dose per gram of tissue (%ID/g).

### Biodistribution

At 2 hours pi, mice were euthanized and dissected. Tumor, inflammation, major organs, and tissues were collected and weighed. The radioactivity of the tissues was measured using a γ-counter. The %ID/g of the tissues was calculated and the results were presented as the mean ± SD.

### Histologic examination and immunohistochemistry (IHC) of PL45 tumors and inflamed muscle

Excised PL45 tumors and the inflammatory thigh muscle were fixed in formalin and embedded in paraffin. Sections 3-µm thick were stained with hematoxylin and eosin (HE) and were processed for immunohistochemistry (IHC). Sections of paraffin-embedded tumor tissues or inflammatory muscles were baked in an oven at 65 °C for 2 h, dewaxed in dimethylbenzene twice, and dehydrated in deionized water and a gradient of alcohol. Antigens on the sections were retrieved with antigen repair solution, and the endogenous peroxidase activity was eliminated by 3% freshly prepared H_2_O_2_. After blocking in 3% BSA at 37 °C for 30 min, the sections were incubated with adequate diluted Anti-hsp90α antibody (1:150) in a wet box at 4 °C for 12 h, followed by the addition of the secondary antibody. After incubation at 37 °C for 30 min and three washes with PBS, sections were stained with a substrate-chromogen solution for 10 min and counterstained with hematoxylin for 3 min before microscopic observation.

### Statistical analysis

All of the data were presented as mean ± SD. IBM SPSS Statistic 22 software (IBM, Armonk, NY, USA) was used to calculate statistics. The data were analyzed using Student's *t* test, and *P* values less than 0.05 were considered to be statistically significant.

## Results

### Synthesis of NOTA-Dimer-San A, cell immunofluorescence, and bioactivity assay

The macrocyclic chelator NOTA was conjugated to Dimer-San A to yield the NOTA-Dimer-San A cyclodecapeptide. Its purity was over 95%, and mass spectroscopy also confirmed the identity of the product 28.

PL45 pancreatic cancer cells were stained with an anti-Hsp90α antibody or Cy5-labeled biotin avidin system (BAS) and found abundant expression of the targeted protein and their co-localization **(**Fig. 2**)**. PL45 pancreatic cancer cells were incubated with different concentrations of NOTA-Dimer-San A or 17AAG for 72 hours. An MTT assay determined the cell viability, which showed a considerable potency as compared with 17AAG. The IC_50_ of the NOTA-Dimer-San A and 17AAG was 234 and 127 nM, respectively **(**Fig. 3**)**.

### Radiochemistry

^18^F-NOTA-Dimer-San A was labeled using the two-step method within 30 minutes with a 29.59 ± 3.78 % radiochemical yield and a radiochemical purity of > 97%. The analytical radio-HPLC data showed that a radiolabeled peak of the product (^18^F-NOTA-Dimer-San A) at 15.96 minutes was well separated from the peak of free ^18^F at 2.51 minutes **(**Fig. 4**)**. For *in vitro* stability, ^18^F-NOTA-Dimer-San A was incubated with PBS or mouse serum at physiological temperature, 37 °C, for 1 and 2 hours. Based on the HPLC analysis, the stability was presented as the percentage of intact radiolabeled probe. ^18^F-NOTA-Dimer-San A exhibited good stability in PBS and mouse serum at 37 °C with the integrity being > 95% after 2 hours of incubation. The octanol-water partition coefficient (log *P*_octanol/water_) was determined to be 1.12 ± 0.13, indicating that ^18^F-NOTA-Dimer-San A is relatively hydrophobic.

### *In vitro* Cell Uptake Assay

The cell uptake assay of ^18^F-NOTA-Dimer-San A showed that the cell uptake in PL45 cells reached 8.03 ± 0.50% at 90 minutes, but decreased slightly at 120 min. In the presence of excess 17AAG, the cell uptake of ^18^F-NOTA-Dimer-San A in PL45 cells decreased to 4.45 ± 0.73% at 90 minutes (*P* < 0.05) (Fig. 5), suggesting that the binding of ^18^F-NOTA-Dimer-San A to PL45 cells is Hsp90-specific.

### Animal PET/CT image acquisition and statistics

The MicroPET imaging study was performed on athymic nude mice (n = 3) bearing Hsp90-positive PL45 human pancreatic ductal adenocarcinoma xenografts and inflammatory lesions (n = 3) at 1 and 2 hours after ^18^F-NOTA-San A injection. Fig. 6 and Fig. 7 show representative decay-corrected coronal images after administration of ^18^F-NOTA-Dimer-San A. The tumor was clearly visualized as early as 1 hour after injection. After normalization, tumor uptake of ^18^F-NOTA-San A was 4.00 ± 0.88 %ID/g and 5.80 ± 0.94 %ID/g at 1 and 2 hours pi, respectively, whereas the inflamed thigh showed minimal uptake (0.85 ± 0.01 %ID/g, 1.50 ± 0.20 %ID/g) at 1 and 2 hours after injection, respectively. The tracer uptake was also calculated for the liver (13.55 ± 1.48 %ID/g and 12.27 ± 2.45 %ID/g), kidneys (4.6 ± 0.85 %ID/g and 5.3 ± 0.21 %ID/g), and muscle (0.99 ± 0.08 %ID/g and 0.88 ± 0.03 %ID/g) at 1 and 2 hours pi. Thus, ^18^F-NOTA-Dimer-San A showed prominent tumor uptake in contrast to the affected thigh, and the activity accumulation between the two groups had a significantly statistic difference (*P* < 0.05).

### Biodistribution

The biodistribution of ^18^F-NOTA-Dimer-San A was examined at 2 hours pi. The %ID/g of different tissues is shown in Table 1. The biodistribution result was consistent with the quantitative analysis of MicroPET imaging. At 2 hours pi, the PL45 tumor uptake of ^18^F-NOTA-Dimer-San A was 4.87 ± 1.50 %ID/g, whereas the inflammation group was 1.47 ± 0.42 %ID/g, which was significantly lower (*P* < 0.05). The T/I (tumor/inflammation) ratio was 3.60 ± 1.80.

### Histology and IHC

Histologic examination of the excised PL45 pancreatic cancer showed a malignant tumor with pleomorphic and hyperchromatic nuclei (Fig. 8A). IHC staining showed high Hsp90 expression, while its expression in the paratumor muscle was negative (Fig. 8C). Additionally, histologic examination of the muscle specimens excised 24 hours after turpentine injection showed an acute inflammatory reaction with massive infiltration of neutrophils in muscle fibers (Fig. 8B), and its Hsp90 expression was also negative (Fig. 8D).

## Discussion

Early detection of pancreatic cancer has been a long-standing challenge 29-32. Hsp90 is a well-established oncogenic target 33, which is expressed in human pancreatic cancer 6- to 7-fold higher than normal tissues. Ogata et al. examined the localization and overexpression of Hsp90 in pancreatic carcinoma tissue as compared to control tissue (including chronic pancreatitis and normal pancreas tissue) and found that Hsp90 alpha mRNA was elevated in pancreatic carcinoma tissue 15. This laid the theoretical foundation for our hypothesis.

Sansalvamide A and its derivatives are Hsp90 inhibitors, which directly bind to Hsp90 and modulate the binding of Hsp90 with other proteins. The interaction of these inhibitors with Hsp90 is specific 25. Dimer-San A cyclodecapeptide is cytotoxic at nanomolar potency levels in pancreatic cancer PL45 cells. This derivative is the most potent Sansalvamide A derivative and does not share structural motifs with existing drugs on the market 23, 34. As compared to macromolecules, small peptides have distinct advantages, including favorable pharmacokinetic and tissue distribution patterns, good permeability properties, low toxicity and immunogenicity, and flexibility in chemical modification and radiolabeling. These favorable pharmacokinetic characteristics are demonstrated via *in vivo* PET application 35, 36. The purpose of this study was to evaluate the feasibility of imaging pancreatic cancer with ^18^F-NOTA-Dimer-San A PET targeting Hsp90.

As for peptide-based molecular probes, modification and potency are very important characteristics to consider 37. 17-AAG is an Hsp90 inhibitor presently in phase III clinical trials that shares the same binding site with San A and its derivatives 38. In this study, Dimer-San A cyclodecapeptide was modified to constitute NOTA-Dimer-San A. PL45 pancreatic cancer cells were stained with an anti-Hsp90α antibody or Cy5 labeled biotin avidin system (BAS), and we observed abundant expression of Hsp90 and their co-localization **(**Fig. 2**)**. An MTT assay evaluated its bioactivity and allowed us to compare it with 17AAG, which showed a considerable potency at nanomolar levels (Fig. 3**)**. ^18^F-NOTA-Dimer-San A was labeled with a 29.59 ± 3.78% radiochemical yield and a radiochemical purity of > 97% (Fig. 4), and exhibited good stability in PBS, as well as in mouse serum with the integrity being > 95% after 2 hours of incubation at 37 °C. The octanol-water partition coefficient (log *P*_octanol/water)_ was determined to be 1.12 ± 0.13. The Hsp90-positive PL45 cell uptake of ^18^F-NOTA-Dimer-San A was not time-dependent, which may be related to the saturation of the Hsp90 receptor. Its binding could be effectively blocked with an Hsp90 inhibitor (17AAG) **(**Fig. 5**)**.

To evaluate the potential of this probe in the differential diagnosis of pancreatic cancer, we established a Hsp90-positive PL45 mouse tumor model and inflammation model. MicroPET imaging of ^18^F-NOTA-Dimer-San A in PL45 tumor-bearing mice at 1 and 2 hours after tail vein injection showed good tumor-to-background contrast, which was 4.00 ± 0.88 %ID/g and 5.80 ± 0.94 %ID/g, and the inflammatory thigh showed minimal uptake (0.85 ± 0.01 %ID/g and 1.50 ± 0.20 %ID/g) at 1 and 2 hours after injection, respectively **(**Fig. 6 and Fig. 7**)**. The activity accumulation between the two groups was significantly different (*P* < 0.05), and the biodistribution data was consistent with the findings. Moreover, histology and IHC confirmed this discovery. As for tumor xenografts, the excised PL45 pancreatic cancer histology showed a malignant tumor with pleomorphic and hyperchromatic nuclei (Fig.8A). IHC staining showed high expression of Hsp90, whereas its expression in the paratumor muscle was negative (Fig.8C). Histologic examination showed an acute inflammatory reaction with massive infiltration of neutrophils in muscle fibers after turpentine injection (Fig.8B) and IHC staining showed negative Hsp90 expression in inflammation (Fig.8D). These results demonstrate the potential this probe has to discriminate pancreatic cancer from inflammation.

It is well known that ^18^F-FDG is a non-specific tracer. Increased glucose metabolism of inflammatory tissues is the main source of false-positive findings in oncology 9. Pancreatic cancer is infamous for its aggressiveness and poor prognosis, and improvements in imaging have the potential to translate into improved patient outcomes by more accurate and rapid diagnosis 5, 39, 40. We previously imaged Hsp90 expression in pancreatic cancer using ^64^Cu-labeled dimeric Sansalvamide A decapeptide, which was measured to be 2.97 ± 0.58 %ID/g at 2 hours and 2.87 ± 0.60 %ID/g at 4 hours post-injection in PL45 tumor mouse xenografts. The accumulation was successfully blocked by Hsp90 inhibitor 17AAG, which confirmed its binding selectivity to Hsp90 28. ^18^F-NOTA-Dimer-San A is a novel probe, which has the potential to discriminate pancreatic cancer from inflammation. Our findings showed that it selectively accumulated in pancreatic cancer tissues, and the inflammatory tissue showed minimal uptake. The IHC result confirmed the imaging findings. Additionally, ^18^F-NOTA-Dimer-San A was more stable, showed higher tumor accumulation, and less liver uptake (log *P* value was determined to be 1.12 ± 0.13, which is better than ^64^Cu-Di-San A1) 28. However, the uptake of ^18^F-NOTA-Dimer-San A in liver is too high, which is possibly related with the hydrophobic properties of the tracer. To further improve the pharmacokinetics of ^18^F-NOTA-Dimer-San A, an appropriate linker, such as PEG units, could be incorporated to prove its water solubility in our next work.

## Conclusion

Dimer-San A cyclodecapeptide, a potent Hsp90 inhibitor, was labeled with ^18^F and successfully converted into a PET molecular probe. It can be concluded that ^18^F-NOTA-Dimer-San A is a novel molecular probe targeting Hsp90, which allows non-invasive imaging of tumor-associated Hsp90 expression. This probe has potential value to distinguish pancreatic cancer from inflammatory masses.

## Figures and Tables

**Figure 1:** The chemical structure of NOTA-Dimer-San A and synthesis scheme for 18F-NOTA-Dimer-San A.

**Figure 2:** ** Confocal immunofluorescence of PL45 pancreatic cancer cells.** The green cells were stained with anti-Hsp90α antibody (B), the red cells were stained with Dimer-San A peptide conjugated with near infrared fluorescence (D), and the blue nuclei were stained with DAPI (A). The final was the merged imaging (C). This image confirmed that Hsp90 was highly expressed in the PL45 cells and that the Dimer-San A peptide bound to the Hsp90 target. Magnification ×60; scale bar = 20 µm.

**Figure 3:** The cell viability (%) and half maximal inhibitory concentration (IC_50_) of different concentrations of NOTA-Dimer-San A decapeptide or 17AAG incubated with PL45 cells for 72 hours. The IC_50_ of NOTA-Dimer-San A and 17AAG was 234 and 127 nM, respectively.

**Figure 4:** The analytical radio-HPLC data shows that the radiolabeled ^18^F-NOTA-Dimer-San A is achieved with a radiolabeled peak at 15.96 min, which is well separated from the peak of free ^18^F at 2.51min.

**Figure 5:** Binding% of ^18^F-NOTA-Dimer-San A to Hsp90-positive PL45 cells with and without blocking reagent (P < 0.05).

**Figure 6:** The representative tumor-bearing mouse model and coronal MicroPET images of ^18^F-NOTA-Dimer-San A in PL45 tumor nude mice (n = 3/group) at 1 and 2 hours post-injection. The images demonstrate great tumor accumulation. Tumors are indicated by red arrows.

**Figure 7:** The representative inflammation-bearing mouse model and MicroPET ^18^F-NOTA-Dimer-San A images at 1 and 2 hours post injection (n = 3/group). The inflammatory lesions are indicated by red arrows.

**Fig 8:** Histology and IHC. PL45 pancreatic cancer showed a malignant tumor with pleomorphic and hyperchromatic nuclei **(A)**. IHC staining showed high expression of Hsp90 (red arrow), whereas its expression in the paratumor muscle was negative (black arrow) **(C)**. Histologic examination of the induced inflammatory muscle specimens showed an acute inflammatory reaction with massive infiltration of neutrophils (black arrow) **(B)**, and its Hsp90 expression was also negative **(D)** (hematoxylin and eosin; Magnification ×20, scale bar = 50 µm).

**Table 1:** Decay-corrected biodistribution of ^18^F-NOTA-Dimer-San A at 2 hours post-injection

Tissue	^18^F-NOTA-Dimer-San A
Blood	1.82 ± 0.57
Heart	3.23 ± 0.84
Bone	1.85 ± 0.60
Lung	6.61 ± 2.18
Liver (L)	19.2 ± 1.43
Gallbladder	7.38 ± 2.99
Spleen	4.54 ± 1.09
Kidneys (K)	9.08 ± 1.87
Pancreas	2.33 ± 0.21
Stomach	2.34 ± 1.85
Intestine	7.12 ± 4.19
Muscle (M)	0.94 ± 0.41
Tumor (T)	4.87 ± 1.50^ a^
Inflammation (I)	1.47 ± 0.42
**Tumor-to-normal or inflammation tissue uptake ratio**	
T/M	5.85 ± 1.69
T/L	0.25 ± 0.07
T/K	0.54 ± 0.11
T/I	3.60 ± 1.80

*P* < 0.05 as compared to the inflammation group.
